The article "The acceptability of using IUDs among Egyptian nulliparous women: a cross-sectional study" was retracted in 2025. Reasons: original data or images not available; unreliable results or conclusions; lack of ethics approval or compliance; concerns about the data.

# The acceptability of using IUDs among Egyptian nulliparous women: a cross-sectional study

**DOI:** 10.1186/s12905-020-00977-9

**Published:** 2020-06-05

**Authors:** Reham Refaat Elkhateeb, Eman Kishk, Ahmad Sanad, Haitham Bahaa, Abdel Rahman Hagazy, Kareem Shaheen, Enas Moustafa, Hahem Fares, Khalid Gomaa, Ahmad Mahran

**Affiliations:** 1 Obstetrics and Gynecology, Faculty of medicine Minia University, Maternity Hospital Minia University, Minia, Egypt; 2 Obstetrics and Gynecology, Faculty of Medicine Suez Canal University, Suez, Egypt; 3 Obstetrics and Gynecology Minia University, Minia, Egypt; 4 Obstetrics and Gynecology, Faculty of Medicine Minia University, Minia, Egypt; 5 Obstetrics and Gynecology at Maternity Hospital, Minia University, Minia, Egypt

**Keywords:** IUD, Nulliparous, Physicians, Attitude towards IUD insertion, Acceptability

## Abstract

**Background:**

Although intrauterine contraceptive device is highly effective, safe, long term and reversible method of contraception, the general population and physicians refuse. IUDs for nulliparous women due to persistent rumors about its side effects and complications. The aim of this study was to assess the acceptability of IUD use in nulliparous women by both women and health care providers in Egypt.

**Methods:**

Five hundred thirty nulliparous women and 200 physicians were interviewed in 10 family planning clinics in Suez and Minia cities – Egypt. The knowledge and attitudes of women and health care providers towards IUD use in nulliparous women were assessed through a well designed questionnaire over 2 years. Those women who accepted using IUD were then followed up for 6 months.

**Results:**

Most of nulliparous women sought for contraception reported a negative impression of IUD method (96.2%). 82.5% of physicians had the same attitude. The reasons for refusing IUD among nulliparous women are fear of side effects including infection (52.8%), and bleeding (37.7%).Also, fear of subsequent infertility 51.9% of women. Regarding the providers, increased pelvic inflammatory disease (PID) represented the highest percentage (70%) for non acceptability, followed by difficult insertion (52.5%). Ninety women who accepted use IUD were followed up 6 months later, 94.4% were still using the method and77.8% were happy with the results.

**Conclusion:**

The main barriers that hinder the use of IUD in nulliparous women are the women insufficient knowledge and attitude of their physicians. Good client counseling. Good training for physician to improve their experience would help increase the use of such effective and safe method.

## Background

In Egypt, contraception is used by up to 57.5% of women in the reproductive years, nearly one third (33.1%) use intrauterine contraceptive devices (IUDs) [1]. IUD has excellent characteristics (high efficacy and safety) making it convenient for use by the majority of women including nulliparous [2]. However, general population and physicians refuse IUDs for nulliparous women due to myths about its side effects and complications. Therefore; IUDs are almost exclusively used by parous women. The exact rate of IUD use in nulliparous women is difficult to ascertain. The acceptability of a contraceptive method is usually inferred from its prevalence of use and method continuation rates. The limited use IUD as a contraception in nulliparous women may be attributed to insufficient counseling by healthcare provider and multiple misconceptions such as the increased risk of pelvic inflammatory disease (PID) and painful insertions [3, 4]. World Health Organization (WHO) guidelines stated that IUDs fall under category two “A condition where the advantages of using the method generally outweigh the theoretical or proven risks” [5]. Previous studies also proved safety and reliability of IUD use in nulliparous women [6, 7]. The 2004 Canadian Contraception Consensus recommended use of IUDs as a contraceptive option for both nulliparous and multiparous women [8]. Now there is evidence that there is no increased risk of PID or infertility in nulliparous women who use IUDs [4, 9].

The article "The acceptability of using IUDs among Egyptian nulliparous women: a cross-sectional study" was retracted in 2025. Reasons: original data or images not available; unreliable results or conclusions; lack of ethics approval or compliance; concerns about the data.

It is hypothesized that there is lack of proper knowledge about IUD use in nulliparous women in Egypt. The aim of this study is to assess the acceptability of IUD use among Egyptian nulliparous women and healthcare providers.

## Methods

A cross-sectional study conducted at 10 public family planning clinics in Suez and Minia cities, Egypt. The clinics were randomly chosen, the closed envelop was the method of randomization. A total of 530 nulliparous women seeking contraception and 200 Physicians from the public clinics were interviewed using a well structured questionnaires. Pilot study was conducted on 30 cases and 20 physicians prior to implementation of the full study. In the pilot study,the provisional study questionnaire was strictly adhered to the complete version of the main study. An important factor measured whether the questionnaire items accurately addressed the research questions. The pilot study tested whether the questionnaire was appropriate, the questions were clearly understood,well defined and presented in consistent manner. All patients and physicians comments were taken into consideration and errors amended till we are sure that there were no further necessary changes. Validity of the questionnaire was tested by sending it to an experts to look at and examine how well designed to measure the concept of the study. The study was approved by ethical committee board of Obstetrics and Gynecology department of both Minia and Suez canal Universities. An informed written consent was obtained from all participants. These family planning clinics were chosen randomly and represented the five areas of the Suez governorate out of seven (Al-Arbeen – El-Suez – Feisal- Ataka – El-Ganayen) and five areas of MiniaGovernorate out of nine (Minia –Mallwi-Abu korkas-Matay–Beni Mazar). Inclusion criteria: for clients All nulliparous women seeking for contraception during the study period, age between 15 and 35, patient approval, able to understand and reply questions during interview in the previously mentioned family planning clinics). Exclusion criteria for clients: Any contraindication for IUD insertion.

The article "The acceptability of using IUDs among Egyptian nulliparous women: a cross-sectional study" was retracted in 2025. Reasons: original data or images not available; unreliable results or conclusions; lack of ethics approval or compliance; concerns about the data.

### Inclusion criteria for physician

All doctors provide contraception services in the previously mentioned clinics, doctor approval to answer questionnaire, MOH training for Cu IUD insertion after graduation, at least 120 patients seen /month, availability of Cu IUD and other contraceptive facilities in their clinics (oral combined .pop, implanol, injectable and barrier methods.) We used two questionnaires; one for women and the other for healthcare providers (physicians). The questionnaires assessed the acceptability of women and physicians to IUD use in nullipara, and barriers that hinder its use in this group. The response rate was 100% for completing the questionnaires (for both women and physicians) for all questions. That is because we have an expert researchers who interview both (women and physician) in a friendly way with maintaining their confidentiality. Questions to assess the acceptability of IUDs in nulliparous women were grouped to cover the following topics: knowledge about the method, viewpoints, anticipated side effects, the effects of the experience of peers and the views of the physician. Open ended questions were used with encouragement to obtain more detailed answers. All questions were simplified and lay person language was used to help women to understand and cooperate. Women were interviewed in privacy and total respect was given to their answers to encourage them to reveals all their concerns. The demographic data of participants were recorded. Providers (physicians) were asked about their knowledge and attitude towards IUDs use for nulliparous women. For physician who refused using IUDs in nulliparous, the reason(s) from the physician’s point of view was mentioned. All data were collected between May 2015 and April 2017. Only Ministry of Health clinics were included because it is serving more than 50% of users. The ministry sent authorization letters in advance of data collection to clinics participating in the study.

The article "The acceptability of using IUDs among Egyptian nulliparous women: a cross-sectional study" was retracted in 2025. Reasons: original data or images not available; unreliable results or conclusions; lack of ethics approval or compliance; concerns about the data.

In cases where the use of IUD in nulliparous women was accepted by women or healthcare providers, no further questions were asked. If there is any concern about its use, women or healthcare providers were given enough time to express their concern in detail then questions were asked to analyze their concerns and to know whether they have any other concerns. All answers were reported in the questionnaire form.

Some women – after good counseling opted for IUD insertion. IUDs (Copper T 380A) were either inserted on the same day or scheduled at a later date. Phone numbers – including mobile and home numbers – were obtained for follow up to check satisfaction, side effects and continuation rate for the use of IUD.

### Statistical analysis

Microsoft Excel 2010 (Microsoft Corporation New York, New York, USA) was used to analyze data. Data were statistically described in terms of frequencies (number of cases) and percentages.

## Results

Five hundred and thirty women were interviewed. The mean age of women involved in the study was 22.35 ± 8.21 years and their characteristics concerning the age groups, educational level and occupation are listed in Table 1. The youngest age group (16–20 years) represented over half of the recruits (54.7%) and most of them were students (51%). Over 90% of women had some form of education. Eighty six physicians (43%) had more than 5 years’ experience in the field of contraception (Table 1). Table 2 shows that - among nulliparous women and physicians – most of them refused IUDs (96.2 and 82.5% respectively). The reasons for refusing IUD among nulliparous women are listed in Table 3 and they included fear of side effects including infection (52.8%), and bleeding (37.7%).Also, fear of subsequent infertility was a significant reason stated by 51.9% of women. Regarding the providers, increased pelvic inflammatory disease (PID) represented the highest percentage (70%) for non-acceptability, followed by difficult insertion (52.5%) as shown in Table 3. Ninety women after good counseling accepted to use IUD and had it inserted. They were quite satisfied with the insertion process (88.9%) and there were minor medium-term complications/side effects; mainly abdominal pains and heavy bleeding. Six months post insertion, most women were still using the IUD (94.4%) and the majority (77.8%) was satisfied with it and would recommend it to another woman (Table 4).

**Table 1:** Characteristics of women and healthcare providers involved in the study

Participants(530) Physcian (200)	Minia		Suez Canal		*P* value
	N	%	N	%	
Age in years					
16–20	155/280	55.4	137/250	54.8	0.83
21–25	65/280	23.3	55/250	22	
26–30	27/280	9.6	23/250	9.2	
> >30	33/280	11.8	35/250	14	
Level of education					
illetrate	28/280	10	17/250	6.8	0.72
primary	97/280	34.6	80/250	32	
secondary	95/280	34	81/250	32.4	
hiegher	60/280	21.4	72/250	28.8	
Occupation					
student	139/280	46.6	118/250	47.2	0.77
housewife	61/280	21.8	49/250	19.6	
teacher	33/280	11.9	27/250	10.8	
clerk	18/280	6.4	25/250	10	
sales	13/280	4.6	17/250	6.8	
other	16/280	5.7	14/250	5.6	
Physcian Years of experience					
Less than 5 years	59/102	57.8	55/98	56.1	0.9
More than 5 years	43/102	42.2	43/98	43.9	0.9

The article "The acceptability of using IUDs among Egyptian nulliparous women: a cross-sectional study" was retracted in 2025. Reasons: original data or images not available; unreliable results or conclusions; lack of ethics approval or compliance; concerns about the data.

**Table 2:** The acceptability of IUDs among nulliparous women and healthcare providers (physicians)

	Nulliparous women	Providers
Accepted	20 (3.8%)	35 (17.5%)
Not Accepted	510 (96.2%)	165 (82.5%)
Total	530 (100%)	200 (100%)

**Table 3:** Reasons for non-acceptability of IUDs use among nulliparous women and physicians

Women (510) and Physicians’ (165) views	The studies population	
	N	%
**Women’s Views**		
**Anticipated Side Effects**		
Increased infection	280	52.8%
Increased bleeding	200	37.7%
Increased pain	170	32.1%
**IUD may cause infertility**	275	51.9%
**‘Migration’ of the IUD**	115	21.7%
**The views of the providers**	180	34%
**Experience of peers**	160	30.1%
**Lack of knowledge**	150	28.3%
**Accessibility**	80	15.1%
**Costs**	45	8.5%
**Efficacy**	40	7.6%
**Physicians’ Views**		
**Increased PID**	140	70%
**Difficult insertion**	105	52.5%
**Increased bleeding**	90	45%
**Increased pain**	75	37.5%
**Expulsion**	30	15%

**Table 4:** Follow up of women who agreed to insert IUD (*n* = 90)

	The studies population	
	N	%
**Age Group (Years)**		
16–20	10	11.1%
21–25	45	50%
26–30	25	27.8%
> 30	10	11.1%
**Satisfaction during the insertion**		
Satisfied	80	88.9%
Not satisfied	10	11.1%
**Side effects / complications experienced within 6 months of insertion**		
Heavy bleeding	20	22.2%
Vaginal infection	5	5.5%
Abdominal pains/discomfort	20	22.2%
Expulsion	0	0%
**Still using IUD as a method of contraception after 6 months**		
Yes	85	94.4%
No	5	5.6%
**Overall satisfaction 6 months post insertion**		
Satisfied	70	77.8%
Not satisfied	20	22.2%
**Would you recommend IUD to a nulliparous woman**		
Yes	70	77.8%
No	20	22.2%

## Discussion

The present study showed that the vast majority of nulliparous women and healthcare providers refrain from using IUD as a method of contraception for reasons such as fear of pain, bleeding, difficult insertion, infection/PID and subsequent infertility. The number of nulliparous women seeking contraception in our country is considered low. This reflects several issues including the conservative nature of the society as sex before marriage is not allowed and hence you would not find a woman seeking contraception publicly outside marriage. Second is the social aspect of seeking pregnancy soon after marriage. In specific conditions such as students in secondary schools or higher education, work rules, low income and second marriage, women may use contraceptive method to delay pregnancy for a while. Indeed, in our study young women (54.7%) and students in schools or higher education (51%) represented the main sectors. Anticipated excessive bleeding and pain (37.7 and 32.1%) were significant reasons for non-acceptability of IUDs among nulliparous women as well as physicians (45 and 37.5%) in this study. A recent study by Hall et al., 2016 included 109 nulliparous women, who had (IUD) either Cu T 380A or (LNG-IUS). Users were surveyed after 1, 6, 12 and 18 months of application. Heavy menstrual blood was more significant in Cu T IUD than LNG-IUS (74% vs 2%; *p* < 0.0001), the author concluded that IUD is safe and well tolerated in nulliparous women [8]. But Hubacher 2007 reported increased menstrual bleeding and pain were higher in nulliparous than in parous women which increased incidence of removal and discontinuation [10]. In a prospective study of 996 insertions in New Zealand, listed nulliparity as a factor associated with difficult insertion (AOR = 5.19, 95%CI 2.49–10.82).Practitioner-reported difficulty with insertion was also associated with nulliparity (1.98; 95% CI 1.11–3.54); however, 80% of insertions in nulliparous women were rated as “easy” by the inserting doctor. The rate of unsuccessful insertion was 2.3% in women with prior vaginal delivery and 11.2% in nulliparous women (*p* < .001) [11]. While Fleming et al., in their study found that IUD insertion can be more painful for nulliparous women and the insertions more difficult for physicians, so the use of IUDs in teenagers and young women was limited [12]. Saav et al. hypothesized that the difficulty during IUD insertion could be decreased or eliminated with the use of cervical dilating agents, such as misoprostol. However, other studies did not confirm this [13]. However, Brockmeyer et al. conducted a study on nulliparous women and their experience of IUD insertion, satisfaction, and continuation over their first year of use. 60% of women described their IUD insertion pain as similar to the pain of a regular period or minor cramping and 15% experiencing very little to no pain [3]. The risk of developing PID after IUD insertion is less than 1% with absence or low risk of acquiring sexually transmitted disease [14]. Suhonen et al. compared the safety of the IUD to OC including the risk for PID. No case of PID was reported in either the IUD group or the OC group [15]. Wiebe et al., 2010 asked 44 nulliparous women who had an IUD inserted within the previous 6 months to report their feedback, almost all of the women were completely satisfied with their choice of IUD [16]. IUD expulsion in the nulliparous population is wrongly believed to be greater in comparison to the parous population, and this has been found to be false. Otero-Flores et al. found the expulsion rate of IUDs in nulliparous women to be less than the parous population [17]. Among all women, particularly those nulliparous, future fertility is an important issue. For many years, IUD insertion and use were suspected to be associated with an increase in the occurrence of PID, leading to possible tubal pregnancy or infertility [18]. In a study by Doll et al., return to fertility within 1 year as not different in women using a barrier method, an oral contraceptive pills or copper IUD [19].

The article "The acceptability of using IUDs among Egyptian nulliparous women: a cross-sectional study" was retracted in 2025. Reasons: original data or images not available; unreliable results or conclusions; lack of ethics approval or compliance; concerns about the data.

The healthcare provider should be aware of WHO and the American College of Obstetrics and Gynecology recommendations [20], and be oriented with new evidence-based information regarding contraception. A cross-sectional survey of 701 healthcare providers was conducted to assess their knowledge related to IUD’s risks, benefits, and uses. The study showed a direct correlation between the time since a provider had graduated from medical school and their knowledge, possess related to IUD use in the nulliparous population [21].

The strengths of the current study are the large number of women and healthcare providers included in the questionnaire, addressing an important untouched issue and potential impact of the study outcome on research and clinical practice. The limitations of the study are conducting the questionnaire in only two governorates from 26 governorates in Egypt and the limited items used in the questionnaire without extending the questions to reveal the source of rumours and misconceptions about the use of IUD in nulliparous women.

The study has implications on both research and clinical practice. Regarding research, it elucidated the need for further large scale questionnaire to be conducted all over the country and involve larger number of women and healthcare providers to know all the misconceptions and rumours about different contraceptive methods. On the clinical practice side, it urges the need for proper training of healthcare providers who are involved in the contraceptive service and improvement of the methods of counselling of women seeking contraception.

## Conclusion

This study concluded that despite the safety, effectiveness and availability of IUD in nulliparous women, it is not being utilised by the general population and physicians in Suez city and Minia Egypt. Women and providers lacked basic and new knowledge of this method,but change physician experience and good counseling of that group would help increase the use of such effective method. However further evaluation and assessment is required.

The article "The acceptability of using IUDs among Egyptian nulliparous women: a cross-sectional study" was retracted in 2025. Reasons: original data or images not available; unreliable results or conclusions; lack of ethics approval or compliance; concerns about the data.

## Data Availability

All data are available upon request from Hossam Shawki head of department of Obstetrics & Gynecology (hossam20012003@yahoo.com) in faculty of medicine, Minia University.

## Abbreviations

IUD: Intrauterine device
Cu IUD: Copper intra uterine device
LNG-IUS: Levonorgestrel intrauterine system
POP: Progesterone only pills
MOH: Ministry Of Health
COC: Combined Oral Contraception
